RETRACTED

# Liquid-Phase Synthesis of Nano-Zinc Oxide and Its Photocatalytic Property

**DOI:** 10.1155/2022/6977424

**Published:** 2022-06-23

**Authors:** Rong Wang

**Affiliations:** Gingko College of Hospitality Management, Chengdu, Sichuan 611743, China

## Abstract

To solve the problem of liquid-phase synthesis of nano-ZnO, a photocatalytic performance study was proposed. In this study, the microwave homogeneous precipitation method was used to add different types and amounts of surfactants. The synthesis of nano-zinc oxide was controlled by changing the reaction system conditions. The photocatalytic properties of nano-zinc oxide for degrading three water-soluble dyes were preliminarily studied and discussed. The results show that the photocatalytic performance of nano-ZnO is closely related to its size, morphology, specific surface area, and even crystallographic direction.

## 1. Introduction

Nanotechnology is one of the most advanced technologies in the world. Nanomaterials science is an interdisciplinary science integrating condensed matter physics, colloid chemistry, coordination chemistry, chemical reaction kinetics, and surface and interface chemistry. Because of their special structure, nanomaterials have many special properties that ordinary materials do not have. Nanomaterials have a wide application prospect in many fields. Compared with ordinary zinc oxide as a functional material, nano-zinc oxide has a series of new special properties in light, electricity, magnetism, chemistry, and biology due to its unique surface effect, small size effect, quantum size effect, and macroscopic quantum tunneling effect. At present, many researches on ZnO nanoparticles have been carried out and great progress has been made in many aspects. Also, many preparation methods of nano-zinc oxide have been successfully investigated. And the application of nano-zinc oxide has also been investigated in the field of photocatalysis, gas sensitivity, and the coating industry, which has achieved great success (Figure 1).

## 2. Literature Review

Because of the surface effect, small size effect, quantum size effect, and macroscopic quantum tunneling effect, nanomaterials exhibit special optical and electromagnetic properties that are different from conventional materials. The unique and novel applications of semiconductor oxides in the fields of light, electricity, magnetism, and catalysis have been paid much attention. Zinc oxide is an oxide semiconductor with a large band gap. When zinc oxide particles reach the nanometer order of magnitude, nanoparticles give zinc oxide many unique and superior properties. By using its wonderful property in light, electromagnetic, and other aspects, the nano-zinc oxide will have remarkable prospects in chemicals, coatings, ceramics, rubber, cosmetics, and other industries [1].

RETRACTED

Bajwa et al. successfully prepared Pt/ZnO hollow birdcage-like special structure by reacting H_2_PtCl_6_ with zinc salt [2]. Harini et al. successfully synthesized petal-like nano-ZnO at low temperature by using zinc sulfate and sodium hydroxide as raw materials and adding cationic surfactants. Nano-zinc oxide from hexagonal granular to a rod and thin film can be successfully synthesized by changing different ratios of mixed solvents of water and ethanol at low temperatures [3]. Ahmed and Makki used the seed growth method of single-crystal Si-coated with Au atom clusters and sapphire substrate to control the growth orientation, preferred growth region, particle diameter, and particle morphology of ZnO nanoparticles [4]. Zhang et al. used Au atom as a catalyst to selectively prepare ZnO nanowire on tungsten substrate and investigated its field emission properties [5].

Nano-zinc oxide is a kind of nanometer material with the most abundant nanometer structure, which has incomparable properties and uses. The morphology, grain size, and distribution of nano-zinc oxide are importantly indexed to measure its properties, which has a particularly significant effect on its properties. Therefore, it is very important to control the grain size, distribution, and morphology of nano-ZnO powder. The controlled synthesis of nano-zinc oxide has aroused researchers' great interest. Various methods are used to regulate the morphology of nano-zinc oxide, to obtain the ideal structure of nano-zinc oxide [6].

## 3. Research Methods

### 3.1. Application Research on Nano-Zinc Oxide

Due to its excellent optical, electrical, chemical, and biological effects, nano-zinc oxide has been widely used in many fields and industries. The functional applications of nano-zinc oxide are shown in Figure 2.

### 3.2. Structure and Properties of Nanomaterials

Nanotechnology refers to the high and new technology that manipulates atoms or molecules on the nanometer scale to produce products with specific functions and studies them to master the laws and characteristics of atoms and molecules. Nanotechnology includes seven areas such as nanophysics, nanomaterials, nanochemistry, nanobiology, nanoelectronics, nanomachinery, and nanomechanics. Nanomaterials, as a branch of nanotechnology, is a new subject that studies the relationship between the composition, structure, and properties of nanomaterials, as well as the preparation, characterization, detection, and application of nanomaterials. Nanomaterials, also known as supramolecular materials, are solid materials composed of ultrafine particles with a particle size between 1 and 100 nm. According to the macroscopic structure, nanomaterials can be divided into nanoblocks, nanofilms, nano-multilayers, and nanofibers. According to the material structure, nanomaterials can be divided into nanocrystals, nanocrystals, and nanocrystals. According to the spatial morphology, it can be divided into zero nanometer particles, one nanometer lines, two-dimensional nanofilms, and three-dimensional nanoblocks [7]. A nanometer is one-billionth of a meter long, the length of three to five atoms packed tightly together. The size of nanomaterials is larger than atoms and molecules, but smaller than ordinary bulk materials. They are in the intermediate field between the microscopic system and macroscopic system, which is called the mesoscopic field. They have four effects that traditional solid materials do not have.

RETRACTED

### 3.3. Small Size Effect

When the size of the component phase of nanomaterials decreases, the properties of the materials change. When the size of the nanoparticles is equal to or less than the wavelength, de Broglie wavelength, and coherence length of the superconducting state, the crystal lattice of the periodic potential field boundary conditions will be destroyed and the quasi-continuous level will be divided into discrete energy levels. The density of atoms near the surface of the amorphous nanoparticles decreases. The acoustic, thermal, optical, electrical, magnetic, and other properties of materials will have new changes, such as the magnetically ordered state to the disorder state and melting point reduction. Such changes are called a small size effect, also called a volume effect. This effect opens up a wide new field for the application of nanomaterials. Using the small size effect of nanoparticles, microwave absorption nanomaterials with a certain bandwidth can be prepared, which can be used for electromagnetic wave shielding, stealth aircraft, etc. [8].

### 3.4. Surface and Interface Effects

Surface and interface effects refer to the change in properties caused by the sharp increase in the ratio of atoms to total atoms on the surface of nanoparticles with the decrease of particle size [9]. As the surface area increases, the particle surface energy and surface tension also increase. There are a lot of atoms on the surface lacking adjacent atoms around. There are many empty suspended bonds, with an unsaturated nature. It is easy to combine with other atoms and tends to be stable, so it has high chemical activity. The specific surface area of spherical particles is inversely proportional to their diameter. And the specific surface area increases significantly with the decrease of particle diameter [10]. The relationship is shown in Table 1.

RETRACTED

It can be seen that as the particle size decreases, the number of atoms on the surface increases rapidly, which is caused by the small particle size and the sharp increase of the surface area. With a large specific surface area, the particles have high surface activity and are easy to combine with other atoms. Using the characteristics of surface activity, metal ultrafine particles are expected to become a new generation of efficient catalysts and hydrogen storage materials [11].

### 3.5. Structure of Nanometer Zinc Oxide

Nano-zinc oxide (ZnO) is an important direct wide band gap semiconductor oxide material, with a band gap of 3.37 eV, exciton binding energy up to 60 meV, and optical gain coefficient of 300 cm^−1^ at room temperature. Nano-zinc oxide (ZnO) crystals have three kinds of structure. The most common is the wurtzite structure, which belongs to the hexagonal crystal system and is a polar crystal. In the ZnO crystal structure, Zn atoms are arranged in close hexagonal packing, and there are four oxygen atoms around each Zn atom, forming a Zn-O4 coordination tetrahedron structure. The surface of the tetrahedron is parallel to the positive plane C (0001). Zn atoms are not symmetrically distributed in the C-axis direction and tend towards the plane [12] (Table 2).

As a new kind of functional material, zinc oxide has excellent ultraviolet shielding, bactericidal and mildew resistance, and electrical properties. At the same time, ZnO is also the only known material with dual characteristics of semiconductor and piezoelectric, which has a very broad development space in energy conversion, especially in micro/nano electronic devices and micro/nano power supply. As the size of nano-ZnO is between atomic clusters and macroscopic particles, it has many special properties that macroscopic materials do not have, and it shows attractive application prospects in many aspects such as electricity, magnetism, chemistry, light, and sensitivity [13].

### 3.6. Research Progress on Preparation Methods of Nano-Zinc Oxide

With further research on the properties of nanometer ZnO powder, many methods to prepare nanometer ZnO powder materials have appeared. According to the state of materials, it can be divided into the solid-phase method, liquid-phase method, and gas-phase method. Each method has its own characteristics, but in general, it develops in the direction of low cost, simple process, high purity, stable size, and few control factors [14].

Solid-phase method, also known as the solid-phase chemical reaction method, is a cheap and simple new method developed in recent years. It is the two substances that were ground, mixed, and then fully ground to get the precursor. And ZnO nanoparticles are finally obtained by heating and decomposition. The raw materials for the preparation of nano-ZnO by the solid-phase method are oxalic acid and zinc acetate or zinc nitrate and sodium hydroxide. ZnC_2_O_4_H_2_O is formed from the former by a solid-state reaction, which is then heated at 460°C and decomposed completely to obtain ZnO with an average particle size of 20 nm. After the latter reaction, Zn(OH) _2_ is obtained, and the size of the calcined product ranges from 20 to 50 nm. The solid-phase method overcomes the disadvantage of particle agglomeration in the traditional wet method and has the advantages of no solvent, high yield, and easy-to-master reaction conditions. However, the reaction process is often incomplete or liquefaction may occur in the process [15].

RETRACTED

The liquid-phase method has incomparable advantages in material preparation, with low production cost, low growth conditions, simple device, easy operation, small particle size, and others, but the use of organic solvents lower the ZnO purity. Common chemical methods for preparing nano-ZnO include precipitation method, sol-gel method, hydrothermal method, microemulsion method, etc. [16].

Vapor deposition is divided into physical vapor deposition (PVD) and chemical vapor deposition (CVD). Physical vapor deposition uses high-temperature heat sources such as electric arc, high frequency, laser, or plasma to heat oxides, vaporize them, and then aggregate them into nanoparticles. Vacuum evaporation (heating under vacuum conditions) is the most commonly used method. Chemical vapor deposition uses volatile metal compounds or metal elemental vapors to generate required compounds through chemical reactions, mainly including gas-phase oxidation and gas-phase pyrolysis [17].

Gas-phase oxidation is the formation of metal oxides by evaporation of metal elements or oxidation reaction of metal compounds in the gas phase. And the vapor of metal oxides condenses into nanoparticles under certain conditions. Nano-ZnO powder synthesis can be obtained by Zn vapor oxidation in an oxygen atmosphere. For example, the research group of Professor Xie Changsheng from Huazhong University of Science and Technology used laser and high-frequency induction double heat source heating methods to evaporate Zn blocks, as shown in equation (1). Nanoscale ZnO and doped nano-ZnO powder were prepared in an oxygen atmosphere and put into actual production [18].

(1) $$\begin{array}{c} \text{Zn}\left(\text{g}\right)+{\text{O}}_{2}⟶\text{ZnO.} \end{array}$$

Gas-phase pyrolysis is to heat the reaction zone to the required temperature with a variety of high-temperature sources in a vacuum or inert atmosphere and then import the gaseous reactants or the reactant solution into the spray method. The solution volatilizes under high-temperature conditions and produces oxides through a thermal decomposition reaction.

RETRACTED

The surface of ZnO nanoparticles prepared by the gas-phase method is clean and the particle size is generally in the range of 10–100 nm. The morphology of ZnO nanoparticles prepared by the gas-phase method is different. So far, its special forms include nano-cantilever ZnO, nano-peg and nano-bridge, nanowire, nanoribbon, nano-ZnO hierarchical structure, etc. [19].

### 3.7. Photocatalysis of Nano-Zinc Oxide

Photocatalysis is the organic combination of photochemistry and catalyst, so light and catalyst are the necessary conditions for triggering and promoting photocatalytic redox reactions. And according to the different substances absorbing photons, photocatalysis can be divided into two types: direct photocatalysis and sensitized photocatalysis. Sensitized photocatalysis refers to the process in which the sensitized agent adsorbed on the surface of the semiconductor absorbs photons under the irradiation of light and is activated, and then the activated electrons are transferred to the semiconductor, causing the oxidation-reduction reaction. Direct photocatalysis refers to the process in which semiconductor molecules are excited and activated after absorbing photons under the irradiation of light, and then a redox reaction occurs with adsorbent molecules. At present, n-type semiconductor oxides are the most widely used photocatalysts. And the photocatalysts investigated include TiO_2_, ZnO, WO_3_, CdS, SnO_2_, Fe_2_O_3_, In_2_O_3_, and so on. TiO_2_ is generally regarded as the best photocatalyst. It is not only nontoxic, harmless, and extremely stable but also very effective in water-phase, gas-phase, and non-aqueous solvents. Although there are various photocatalysts with different catalytic activities, the photocatalytic principle of compound semiconductors is basically the same, especially ZnO and TiO_2_ semiconductor oxides, which have roughly equivalent wide band gap width and both belong to wide band gap n-type semiconductor oxides [20].

Semiconductor materials can be used as photocatalysts because of their own photoelectric characteristics. The band structure of semiconductor particles is generally composed of the low energy valence band and the high energy conduction band, and there is a gap between the valence band and conduction band [21].

When light with energy greater than or equal to the energy gap (hv ≥ Eg) hits the semiconductor, the semiconductor particle absorbs light and generates electron-hole pairs. Unlike metals, semiconductor particles lack a band connection region. And electron-hole pairs generally have picosecond lifetime, sufficient to allow photogenerated electrons and photogenerated hole pairs to transfer charge via the band gap to materials adsorbed on the semiconductor surface from the solution or gas phase. The overall reaction process of photocatalytic degradation of organic pollutants by semiconductor photocatalyst can be represented by equation (2).

(2) $$\begin{array}{c} \text{Organic}+{\text{O}}_{2}+\text{semiconductor}⟶{\text{CO}}_{2}+{\text{H}}_{2}\text{O}+\text{mineralized.} \end{array}$$

The reaction process can be divided into the following steps.

RETRACTED

The first step is that under the excitation of the light source of a certain wavelength, the electrons can be excited from the valence band to the conduction band. At the same time, corresponding holes are generated in the valence band and the conduction band generates electrons, thus generating electron-hole pair as shown in formula (3).

(3) $$\begin{array}{c} \text{Semiconductor}+\text{hv}⟶\text{hv.} \end{array}$$

The second step is that the semiconductor in an aqueous solution and under the action of an electric field separates the electrons from the holes and migrates to different positions on the particle surface, thus participating in the redox reaction, reducing, and oxidizing the material adsorbed on the surface.

Photoinduced holes have a strong ability to obtain electrons and have a strong oxidation ability. They can capture electrons in organic matter or solvent on the surface of semiconductor particles so that substances that do not absorb light can be activated and oxidized. At the same time, photogenic holes also interact with water to generate hydroxyl radicals with strong oxidation, which can attack most organic compounds without selectivity, as shown in formulas (4) and (5).

(4) $$\begin{array}{c} {\text{h}}_{\text{vb}}+{\text{H}}_{2}\text{O}⟶\text{H}+\text{OH,} \end{array}$$

(5) $$\begin{array}{c} {\text{h}}_{\text{vb}}+\text{OH}⟶\text{OH.} \end{array}$$

The third step is the oxidation of organic matter by strong oxidants with photogenerated holes and hydroxyl radicals, generating organic radicals and then oxidizing into oxygen radicals in the presence of molecular oxygen. These intermediates undergo oxidative degradation through thermodynamic reactions to become water, carbon dioxide, and minerals, as shown in formula (6).

(6) $$\begin{array}{c} {\text{h}}_{\text{gt}}+\text{organic}⟶\text{ organic}+\text{oxidation of organic or OH}+\text{organic.} \end{array}$$

RETRACTED

## 4. Experiment and Research

### 4.1. Liquid-Phase Synthesis Method of Nano-Zinc Oxide

#### 4.1.1. Precipitation

Precipitation is the main method to prepare nano-powder by adding appropriate precipitant to the raw material solution to form corresponding precipitation of cations in the raw material solution. The precipitation method can be divided into the direct precipitation method and uniform precipitation method according to the precipitation mode [22].

#### 4.1.2. Direct Precipitation Method

The direct precipitation method is to add precipitant in soluble salt solution and generate precipitation under certain conditions. Wash and dry the precipitation to get precursors. Precursors are through thermal decomposition to get products. Common precipitators are NaOH, NaCO_3_, NH_3_, H_2_O (NH_4_)_2_ CO_3_, NH_4_HCO_3_, and so on.

Nano-zinc oxide is prepared by direct precipitation method using zinc acetate and ammonium bicarbonate as raw materials with surfactants. The average particle size of zinc oxide is 20∼80 mm and the crystal is hexagonal. Using zinc chloride and ammonium carbonate as raw materials, the influence of the precursor calcination time at 300°C on the particle size of nano-zinc oxide is compared and the optimal preparation process of nano-zinc oxide is obtained [23].

Direct precipitation is used to investigate the effects of different feeding methods on the microstructure of nano-zinc oxide and the precursors of the two methods are characterized, and the kinetic law of nano-zinc oxide grain growth is obtained. Some scholars have investigated the types and concentrations of precipitators and feeding methods and concluded that the size of zinc oxide powder is different with different precipitators and feeding methods also affect the morphology and particle size of products [24].

The direct precipitation method has the advantages of a simple process, low equipment requirements, and low cost. However, the introduction of a large number of anions in the solution requires repeated washing, and there are shortcomings such as a long technological process, difficulty to clean waste liquid, and poor dispersion of materials [25].

#### 4.1.3. Uniform Precipitation Method

The uniform precipitation method uses a chemical reaction to make the precipitator evenly release the crystal ions throughout the solution. The precipitant added does not immediately react with the precipitated component. Instead, a chemical reaction causes the precipitant to form slowly throughout the solution. Common uniform precipitators are urinary cord and hexamethylenetetramine. Nano-zinc oxide powder was synthesized by a uniform precipitation method with zinc nitrate as raw material and urea as precipitant. Nano-zinc oxide particles are hexagonal crystal system. The particle size is about 50 nm. In the mixed solvent of ethanol and water, various morphologies of zinc oxide are prepared by adjusting the reaction conditions such as reactant concentration and heating mode. Using zinc nitrate as raw material, hexamethylenetetramine as precipitator and surfactant polyacrylamide diallyldimethyl ammonium chloride (PAM-CTAC) as a morphology control agent, zinc oxide nanorings with an inner diameter of 220 nm and wall thickness of 70 nm are synthesized by uniform precipitation method at low temperature. Through the research, the key role is PAM-CTAC. Changing the concentration of PAM-CTAC can effectively achieve a controllable synthesis of zinc oxide nanoring. Nano-zinc oxide is prepared by a uniform precipitation method. The effect of surfactant on particle size and morphology of the product is investigated.

RETRACTED

The particles of the precipitate obtained by the uniform precipitation method are uniform and compact, which is convenient for filtering and washing and can avoid the co-precipitation of impurities. The product distribution is narrow and the dispersion is good. However, the uniform precipitation method for the preparation of nano-zinc oxide technology is harsh and the reaction time is long.

### 4.2. Research on Photocatalytic Property of Nano-Zinc Oxide

The photocatalytic activity of ZnO nanoparticles with different morphology and grain size is also changed with morphology and crystallization degree. The photocatalytic activity of ZnO nanoparticles with different morphologies is different when degrading RhB dye. Among them, the flower-shaped nano-ZnO has the highest photocatalytic activity. In the process of photocatalytic degradation, the amount of catalyst, pH value of the solution, initial concentration of dye solution, and light intensity have important effects on the photodegradation reaction.

The photocatalytic degradation of three water-soluble dyes wastewater by nano-ZnO prepared with cationic surfactants cetylpyridine chloride and cetyltrimethyl ammonium bromide is investigated. The preparation of nanometer zinc oxide by two kinds of cationic surfactants on three different decoloring degradation rates of water-soluble dyes are examined. By the UV-Vis spectrophotometer method, the dye molecules in the aromatic ring structure in the process of degradation decoloring are analyzed. The different types and different dosages of surface-active agents on the properties of nanometer zinc oxide photocatalytic effect are compared.

### 4.3. Test Method

About 100 mL of three dye solutions with a mass concentration of 12 mg/L were taken into a 250 mL beaker and a certain amount of self-made nano-zinc oxide was added. After being stirred evenly and fully adsorbed in a dark place, the photocatalytic degradation experiment was carried out in an indoor environment with no light and a UV lamp (20 W, wavelength 254 nm), and a blank control test was conducted. After centrifugation, the absorbance of the sample was measured by UV-Vis spectrophotometer at the maximum absorption wavelength of the dye. The degradation rate was calculated according to *a* = (1 − *A*/*Ao*) × 100%, in which *A* and *Ao* were the absorbance of the organic dye solution at the maximum absorption peak, respectively.

RETRACTED

### 4.4. Experimental Results

Since the concentration value of dye solution in the range of low concentration is linear with the absorbance value, the absorbance can be used to represent the content of dye indirectly. So, the formula of the photocatalytic degradation rate is (C − C)/Co. The plot with C/Co as ordinate and photocatalytic time *t* as ordinate can reflect the relationship of degradation rate with time. The experiment results showed that only synergistic action of ultraviolet irradiation and zinc oxide catalyst happened, the three water-soluble dyes could be degraded well. Among them, the acid magenta was the most easily degraded, and the degradation rate could reach 99% after 2 hours. Both products A1 and A3 could completely catalyze the degradation of dyes in a short time, with good catalytic activity, and the catalytic activity decreased with the increase of particle size. The photocatalytic degradation rate of dyes by ZnO nanoparticles prepared with different surfactants was obviously different. The degradation rate of product A1 was poor and that of product A3 was good. And their degradation rate was different with different dyes. According to the above experimental results, the morphology and particle size of nano-zinc oxide particles prepared under microwave conditions were different with the addition of different kinds or different concentrations of cationic surfactants, and the morphology and particle size strongly affected the activity of the photocatalyst. The main reason was that nanoparticles were with quantum size effect. As the particle size was smaller by a certain value, the conduction band and valence band were changed into discrete energy levels. The energy gap grew wider. The valence band became more positive and the conduction band became more negative. The redox ability of electrons generated by light and holes increased, improving the activity of nanometer zinc oxide oxidation of organic compounds. Due to the large specific surface area and a large number of atoms on the surface, the photocatalytic adsorption capacity of zinc oxide was improved. The smaller the radius was, the shorter the diffusion time of photogenerated charge from the body to the surface. The higher the separation efficiency of photogenerated charge was, the lower the recombination rate of electron and hole was, which led to the improvement of photocatalytic activity (Figures 3 and 4).

RETRACTED

The apparent rate constant of photocatalytic degradation and the reaction kinetic equation can be obtained by linear regression to compare the photocatalytic performance of each sample. As can be seen from Table 3, the photocatalytic degradation of dyes by nano-ZnO powder was in accord with first-order reaction kinetics and had good linearity. The reaction apparent rate constant *k* of product A3 degradation acid fuchsin was the highest, indicating that the catalyst had the highest photocatalytic activity and the dye was easily degraded. The degradation rate constant of malachite green was the lowest for product A1 and the dye was the most difficult to degrade. For the same dye, the morphology and size of nano-ZnO photocatalyst were different and the degradation rate was also very different.

The morphology and size of ZnO nanoparticles prepared by different amounts of surfactants were different and their photocatalytic performance was also different. Two prepared products A1 and A3 were used as catalysts and methylene violet was used as the research object to carry out a photocatalytic degradation experiment. The results are shown in Figure 5.

The apparent rate constant and kinetic equation of the photocatalytic degradation of methylene violet dye was obtained by linear regression to compare the photocatalytic performance of each product. For cetylpyridine chloride, with the increase in dosage, the size of ZnO nanoparticles decreased. As the surface area increased, the photodegradation surface became larger and the catalytic activity increased. For cetyltrimethyl ammonium bromide, the slenderness ratio decreased, the morphology changed, and the degradation rate decreased with the increase of concentration. These results indicated that the photodegradation rate of the prepared products to methylene violet was different with the addition of a different amount of surfactant. The photodegradation rate of the prepared product decreased with the increase in the amount of surfactant, which was caused by the increase in the amount of ZnO rod diameter and the decrease of the photodegradation surface. The photocatalytic performance was determined by the synergistic effects of particle size, morphology, specific surface area, and other factors.

## 5. Conclusion

By the microwave homogeneous precipitation method, two kinds of cationic surfactants cetylpyridine chloride and cetyltrimethyl ammonium bromide were added to prepare nano-zinc oxide powder by microcontrol. The morphology of the product was characterized by FT-IR, XRD, and SEM. The morphology and size of the product changed greatly after the surfactant was added. The product ZnO prepared by adding cetylpyridine chloride was long and coarse rod shape with large particle size and regular morphology. With the increase in dosage, the particle size decreased. The product prepared by adding cetyltrimethyl ammonium bromide was granular with a small particle size and the dispersivity of nanometer ZnO prepared by cetyltrimethyl ammonium bromide was better than that prepared by cetylpyridine chloride in ethanol medium. Therefore, different kinds of surfactants played different roles in the preparation process and the selection of surfactants was very important for the preparation of nano-zinc oxide with different morphologies.

RETRACTED

Three water-soluble dyes were used to investigate the photocatalytic property of the products. The results showed that the morphology and size of the products had a great influence on the photocatalytic property and the products with large particle size had poor photocatalytic property. As the particle size decreased, the specific surface area increased and the photocatalytic activity increased. The photocatalytic property was determined by the synergistic effects of particle size, morphology, specific surface area, and other factors.

## Figures and Tables

**Figure 1:** Nano-ZnO and its photocatalytic property.

**Figure 2:** Function of nano-zinc oxide.

**Figure 3:** Degradation of acid fuchsin by-products A1 and A3.

**Figure 4:** Degradation of methylene violet by-products A1 and A3.

**Figure 5:** Degradation curves of methylene violet by the two products.

**Table 1:** The relationship between the size of nanoparticles and the number of atoms on the surface.

Nanoparticles size/m	Total number of atoms contained (*N*)	Percentage of atoms on the surface (%)
90	3 *∗* 10^4^	3
20	3 *∗* 10^6^	21
5	3 *∗* 10^3^	50

**Table 2:** Characteristic parameters of hexagonal fibril ore.

Property	Value	Property	Value
Stability	Wurtzite structure	Band gap	3.39
Melting point/C	2.693	Hall mobility	210
Density/(gcm)	4.256	Effective hole mass	0.58
Refractive index coefficient	1.962	Linear expansion coefficient	6.5 *∗* 10^6^

**Table 3:** Kinetic parameters of first-order reaction for degradation of three dyes.

Product	Degradation of dyes	Reaction kinetic equation	Linear correlation coefficient	Apparent rate constant
A1	Acid magenta Methylene violet Malachite green	*Y* = −0,09762 + 0.98343*X* *Y* = −0.14714 + 0.72000*X* *Y* = −0.11893 + 0.70029*X*	0.9632 0.9563 0.956	0.89 0.59 0.95

A3	Acid magenta Methylene violet Malachite green	*Y* = −0.12238 + 1.18857*X* *Y* = −0.14750 + 1.06786*X* *Y* = −0.19607 + 0.94786*X*	0.998 0.965 0.983	0.36 0.59 0.36

RETRACTED

## Data Availability

The data used to support the findings of this study are available from the corresponding author upon request.
